# A Defect Detection Method for Rail Surface and Fasteners Based on Deep Convolutional Neural Network

**DOI:** 10.1155/2021/2565500

**Published:** 2021-07-29

**Authors:** Danyang Zheng, Liming Li, Shubin Zheng, Xiaodong Chai, Shuguang Zhao, Qianqian Tong, Ji Wang, Lizheng Guo

**Affiliations:** ^1^School of Urban Railway Transportation, Shanghai University of Engineering Science, Shanghai 201620, China; ^2^School of Information Science and Technology, Donghua University, Shanghai 201620, China; ^3^School of Computer and Data Science, Henan University of Urban Construction, Pingdingshan 467036, Henan, China

## Abstract

As a result of long-term pressure from train operations and direct exposure to the natural environment, rails, fasteners, and other components of railway track lines inevitably produce defects, which have a direct impact on the safety of train operations. In this study, a multiobject detection method based on deep convolutional neural network that can achieve nondestructive detection of rail surface and fastener defects is proposed. First, rails and fasteners on the railway track image are localized by the improved YOLOv5 framework. Then, the defect detection model based on Mask R-CNN is utilized to detect the surface defects of the rail and segment the defect area. Finally, the model based on ResNet framework is used to classify the state of the fasteners. To verify the robustness and effectiveness of our proposed method, we conduct experimental tests using the ballast and ballastless railway track images collected from Shijiazhuang-Taiyuan high-speed railway line. Through a variety of evaluation indexes to compare with other methods using deep learning algorithms, experimental results show that our method outperforms others in all stages and enables effective detection of rail surface and fasteners.

## 1. Introduction

In recent years, rail transportation has become one of the most important modes of travel. As the total mileage of rail transit continues to increase, how to ensure safe railway operation has become a dominant issue that has attracted public attention. As shown in Figure 1, the rail is the main component of the railway track and is utilized to guide the wheels of the train forward and bear the pressure of the wheel set. The rail and its fasteners in the service are affected by contact forces such as extrusion and impact of the train wheel-rail, poor environment, and material aging. These problems have led to the continuous deterioration of railways, inducing the formation of rail surface defects such as peeling, collapse, abrasion, and corrosion, as well as fastener defects such as fracture and loosening [1]. Research results show that many rail fractures or train derailments are caused by rail surface or fastener defects. Therefore, it is crucial to ensure that the rail and its fasteners are in a healthy state that maintains the safety and stability of train operation. At present, state detection of the rail and its fasteners on the railway track line is mainly conducted through inspections by railway staff. Although this inspection method has the advantages of simplicity and low cost, it also has disadvantages such as low detection efficiency, high missed detection rate, and poor real-time performance. In recent years, defect detection technology based on computer vision has been widely used in industry [2–6]. Some scholars have begun to employ computer vision technology to detect the defects of rails and their fasteners, so that the problems of manual inspection can be solved.

Using a localization algorithm is necessary to improve the accuracy of defect detection and localize the track components to be inspected, so that the influence of redundant information such as background can be reduced. Commonly used localization methods are template matching [7], pixel statistics [8], and edge detection [9]. However, localization methods of pixel statistics and edge detection are susceptible to uneven lighting and complex backgrounds. The traditional template matching method is difficult to use in localizing deformed or damaged track parts. To solve this problem and localize the track fasteners, Qiu et al. [10] proposed a double-template matching method. First, the rail template is used to localize the rail in the horizontal direction and then use the fastener template to localize the fastener in the vertical direction. In addition, Li et al. [11, 12] used the geometric characteristics of track components to localize fasteners, and Wei et al. [13] used the variance projection and wavelet transform to localize the edges of the rail, fasteners, and backing plates based on the fixed positional relationship between the track components.

The detection method of rail fasteners based on traditional vision mainly uses artificially designed features to extract the features within the fastener area and then inputs the extracted features into a classification model based on shallow learning to classify the state of the fasteners. The shallow features used in the research articles on fastener detection mainly include Haar-like feature [7, 14], Dense-SIFT feature [13], direction field feature [15], edge feature [16], HOG feature [17], Gabor filter feature [18], and Hough transform feature [11, 12]. Classification models mainly include AdaBoost classifier [7, 19], support vector machine (SVM) [17, 18, 20], probabilistic graphical models (PGM) [13], and multilayered perception neural classifier [21, 22]. However, this type of detection method extracts features for the fastener area rather than the detection object. The extracted features are susceptible to the influence of background information, with low robustness and low accuracy for the identification of fasteners in abnormal states. In recent years, as the application of deep learning technology in image processing has achieved great success, many scholars have also begun to try to apply deep learning technology to rail fastener detection. Li et al. [23] used a method based on semantic segmentation algorithm to detect the state of fasteners First, the saliency model is used to localize the track fastener area, and then PSPNet is used to semantically segment the fastener subimages. Finally, the state of the fastener is judged by the vector geometry measurements of the fastener. Gibert et al. [24] used a customized fully convolutional network to extract the highly abstract features of fasteners and identify fastener types and then utilized customized support vector machines to classify the state of fasteners for various types of fasteners. Ma et al. [25] cropped out the bolt area subimages that were not related to the identification of the fastener state on the fastener area image and then used the CNN network for classification. Through this approach, the accuracy rate is improved compared to that with the classification directly in the fastener area. To address the impact of the imbalance problem of the dataset samples on the performance of the detection model, Liu et al. [26] proposed a similarity-based deep network, which obtains a large number of training samples by combining an abnormal sample with multiple normal samples. Liu et al. [27] proposed to use U-Net to generate a large number of defective fastener samples, after which the fasteners were detected using convolutional neural network.

In the last decade, many scholars have conducted research on the detection methods of rail surface defects. These methods mainly solve three problems, namely, the classification of rail surface defects [28, 29], location of rail surface defects [30–33], and pixel-level segmentation of rail surface defects [34–37]. Among them, the pixel-level segmentation of rail surface defects is a key research problem. Nieniewski [34] proposed a detection method based on morphological processing for pixel-level extraction of rail surface defects. The main advantage of this method is the fast detection speed that can reach 50 ms/frame. Yu et al. [35] proposed a three-stage coarse-to-fine model. At the first stage, the background subtraction model is used to filter the images of the defect-free rail surface area; at the second stage, the region extraction model is used to localize the defective area; and at the last stage, a pixel subtraction model is used to detect the defective contours and perform pixel-level extraction. However, this method involves many steps and is sensitive to noise. Niu et al. [36] applied a binocular line-scanning system to the detection of rail surface defects and used global low-rank, nonnegative reconstruction saliency algorithm, and depth outlier detection to combine the two-dimensional saliency map and the three-dimensional defect contour to obtain the final output result. In recent years, there has been a great development of the detection of rail surface defect using deep learning techniques. Faghih-Roohi et al. [38] proposed to use DCNN to classify images of rail surface areas with defects. Shang et al. [39] used traditional object positioning algorithms to localize the rail surface area on the original track image and then used a fine-tuned CNN network to divide the rail surface subimages into two categories: defective and intact. However, the aforementioned two methods did not detect the specific location of the defect. Song et al. [40] used the YOLOv3 network to localize the defect on the rail surface, but this method did not obtain the specific size and shape information of the defect. Liang et al. [41] used the SegNet network to identify and segment the defects, but the segmentation accuracy of this method needs to be improved. James et al. [42] proposed TrackNet, which integrates U-Net and ResNet for defect semantic segmentation and classification, respectively. This method improves the accuracy of defect recognition, but the accuracy of semantic segmentation needs to be improved.

The aforementioned methods are mainly aimed at detecting a single railway track component. However, the track images collected in the railway line usually contain both rails and fasteners. If both are detected at the same time, the detection efficiency can be greatly improved. To the best of our knowledge, only one article considers the defect detection problem of rail surface and fasteners simultaneously. Wei et al. [43] used the improved YOLOv3 model to realize the simultaneous detection of rail surface defects and fasteners in the railway track line image and obtained high detection accuracy. However, the types of fasteners considered in this article are different from those considered in our study. This method cannot detect the specific location and size of the rail surface defects, and the detection speed is difficult to meet the actual needs of the project. Realizing the pixel size detection of the surface defect area of the rail helps the inspector judge the degree of the rail disease. For this reason, we propose a detection method based on convolutional neural network (CNN) to automatically detect the rail surface defects and the state of the fasteners on the railway line, in Figure 2. First, we utilize the improved YOLOv5 framework to localize the rail and fasteners in the original railway track line image. Then, a defect detection model based on the Mask R-CNN is designed to semantically segment the defects in the rail subimages. In addition, the ResNet network is used to classify the fastener state in the fastener subimages into normal, loosening, and broken.

The contributions of this study are summarized as follows:

1. A railway line key component multiobject detection method is proposed based on a series of deep convolutional neural networks, which can achieve the detection of rail surface defects and fastener state.
2. An improved YOLOv5s framework is proposed to localize the rail and fastener in the railway track line image at the same time, and the Ghost bottleneck is used to optimize the backbone network of the original YOLOv5s to effectively reduce the number of parameters and the computational cost. This method can be used for both ballast and ballastless track line image detection. Compared with the original YOLOv5s and other advanced object detection models, the detection speed is significantly improved while maintaining high accuracy.
3. The two-stage object detection algorithm, Mask R-CNN, is used in the detection of rail surface defects, which effectively improves the recognition and segmentation accuracy.
4. A set of state classification criteria for slab fast clip (SFC) type fastener are proposed.

The rest of this article is organized as follows: Section 2 introduces the rail and fastener positioning method based on the improved YOLOv5.  Section 3 describes the rail surface defect detection model based on Mask R-CNN algorithm.  Section 4 introduces the state classification criteria of SFC-type fasteners and the classification model used in this paper.  Section 5 designs comparative experiments with other competitive methods to verify the effectiveness of our method. Finally, conclusions and future work are presented in Section 6.

## 2. Localization of the Rail and Fastener

### 2.1. YOLOv5 Framework

In this study, we use the improved YOLOv5s object detection neural network to localize the rail and fasteners in the original track images collected from the railway site. The network framework is shown in Figure 3.

The You Only Look Once (YOLO) series network is a one-stage object detection algorithm for object localization and recognition in the image. This algorithm extracts image features by CNN and directly calculates the classification score and object localization [44]. Compared with YOLOv3 and YOLOv4, YOLOv5 is optimized for data enhancement, network structure, and loss function. YOLOv5 uses the following data enhancement methods to improve the robustness of the model: mosaic data enhancement, adaptive anchor box calculation, and adaptive image scaling. Both YOLOv5 and YOLOv4 use mosaic data enhancement to improve the detection ability of the model for small objects. Adaptive anchor box calculation can calculate the best anchor box value depending on different training data sets. Adaptive image scaling can improve the speed of object detection by adding a minimum of black borders when scaling the image. In terms of network structure, YOLOv5 adds a Focus component to the Backbone to perform slicing operations on images, retaining more complete image downsampling information for subsequent feature extraction by adding some floating point operations (FLOPs). The Neck Network chose path aggregation network (PANet) [45] to improve the problem of difficult propagation of low-level features of the original feature pyramid networks (FPN) [46] and strengthened the fusion of extracted features. The Head network chose the same as YOLOv3 and YOLOv4 to realize object detection. The loss function of YOLOv5 is mainly composed of three parts, including bounding box loss, classification loss, and confidence loss. The binary cross entropy is used as the loss function of the classification loss and the confidence loss to calculate the category probability and the target confidence score. We use CIoU loss as the loss function of bounding box, which better describes the regression of rectangular boxes [47].

### 2.2. Backbone Optimization

The original YOLOv5 network used cross stage partial (CSP) bottleneck [48] to increase the depth of the network and thus improve the network's ability to extract features. However, in the task of rail and fastener localization, we have found that utilizing some modules with lower computational costs to simplify the structure of the model can also achieve satisfactory experimental results. To facilitate our model to be deployed on some low-performance devices with small memory, such as track inspection vehicles or embedded devices, we used a lightweight Ghost bottleneck [49] instead of the CSP bottleneck in the original network to reduce the size of the model and increase the inference speed of the network, as shown in Figure 4. The core idea of the Ghost bottleneck is to use some cheap cost linear operation to generate many feature maps with rich information. Specifically, first, use a small amount of conventional convolution operations on the feature map to generate intrinsic features, then use some cheap cost linear transformation on the feature map to generate another part of the feature, and finally integrate the two parts together as the final output feature.

The structure of the Ghost bottleneck is shown in Figure 5. Ghost bottleneck consists of two Ghost modules. The network first goes through a Ghost module to increase the number of channels, then a deep-wise convolution to reintegrate the features, and finally a Ghost module to match the number of channels with the shortcut paths. The two are added together to obtain the final output. Ghost module includes convolution operation and linear transform, and its calculation formula is as follows:

(1) $$\begin{array}{c} Y=X*f,\\ y_{\left(i,j\right)}^{,}=\varphi_{\left(i,j\right)}\left(y_{i}\right), \end{array}$$

where *X* is the input data, *∗* is the convolution operation, and *Y*=[*y*_1_, *y*_2_,…, *y*_*i*_,…, *y*_*m*_] is the output data, which means that the *m* channel feature map is obtained after the convolution operation, 1 ≤ *i* ≤ *m*, *φ*_(*i*, *j*)_(*y*_*i*_) in the aforementioned formula is the *j*-th linear transformation of the *i*-th feature map, and  *Y*′=[*y*_(1,1)_′, *y*_(1,2)_′,…, *y*_(*i*, *j*)_′,…, *y*_(*m*, *s*)_′] represents the feature map of *m* × *s* channels obtained by linear transformation, 1 ≤ *j* ≤ *s*.

The Ghost module can flexibly define the number of convolution kernels and enlarge the number of channels of the input feature map by *s* times. Adding a deep-wise convolution between the two Ghost modules can effectively increase the tolerance to changes in the geometric features of the rail and fasteners and reduce the parameter redundancy. Batch normalization (BN) is added after the convolutional layer of each module, and the hard-Swish [50] activation function is added after the convolutional layer of the two Ghost modules to improve the expressive ability of the neural network.

## 3. Rail Surface Defect Detection

In this paper, the Mask R-CNN model is used to localize and segment the defects in the rail surface image.

Mask R-CNN is an improved two-stage object detection network based on the Faster R-CNN framework [51]. On the basis of Faster R-CNN [52], Mask R-CNN optimizes the architecture for bounding box regression and object classification at the first stage and adds the FCN [53] branch for the second stage of predicting segmentation masks. The network structure is shown in Figure 6.

First, the rail surface image is input to the feature extraction network to generate a multiscale feature map. Second, the obtained feature map is input to the region proposal network (RPN) network to generate a region of interest (RoI). Then, the RoI of different dimensions generated by the RPN network is transformed to features of the same dimension by the RoI Align operation. Finally, the obtained features are, respectively, input to the fully connected layer and FCN for rail surface defect classification, bounding box regression, and segmentation mask prediction.

The rail surface defect detection model designed in this study uses Resnet50 [54] +FPN as the feature extraction network. Using Resnet50 can enable extraction of features at different scales on the rail surface image. However, if only Resnet50 is employed as a feature extraction network, there is the problem of weak detection ability of objects with small objects occurs, which can easily fail to detect small defects on the rail surface. Therefore, adding RPN to integrate the low-level and high-level features of Resnet50 can effectively improve the ability of small defect detection. Four different feature maps from P2 to P5 are used in FPN. Depending on the size of the RoI, different scales of feature maps should be selected. It is ensured that large RoIs are generated from high-semantic feature maps, which is conducive to the detection of large defects, and small RoIs are generated from high-resolution feature maps, which is conducive to the detection of small defects. The specific selection formula is

(2) $$\begin{array}{c} k=k_{0}+\;\log_{2}\left(\frac{\sqrt{wh}}{224}\right), \end{array}$$

where *k*_0_=4, *w* and *h* are the width and height of RoI, and *k* is the number of layers of the feature map in FPN. To input RoIs of different dimensions to the fully connected layer for classification score calculation and bounding box regression, transforming RoIs of different dimensions to the same dimension is necessary. Mask R-CNN utilizes RoI Align instead of RoI Pooling in Faster R-CNN. RoI Align uses a bilinear interpolation to obtain the values of multiple sampling points and then uses the maximum pooling of the values of multiple sampling points to obtain the final value of the point. This method effectively solves the position mismatch problem caused by two quantization operations in RoI Pooling and can effectively improve the accuracy of detection or segmentation. Finally, the loss function of Mask R-CNN is

(3) $$\begin{array}{c} L=L_{\text{box}}+L_{\text{cls}}+L_{\text{mask}}, \end{array}$$

where *L*_box_ and *L*_cls_ are the same as in Faster R-CNN [52], representing the bounding box regression loss and object classification loss, and *L*_mask_ is the mask loss. The mask branch in the network uses the Sigmoid function for each pixel on the mask, then feeds it into the cross-entropy loss, and defines the average of all pixel losses as the mask loss.

## 4. Fastener State Classification

### 4.1. Judgment Criteria for Fastener State

The track fasteners used in this experiment are Pandol fast clip. The fasteners in the track images collected on the railway line are in three states, namely, normal, loosening, and broken, as shown in Figure 7. Currently, no set of criteria is available to classify the normal and loosening states of SFC-type fasteners. Therefore, this study divides the fastener area into the two parts shown in Figure 8 as the criteria for judging the state of the SFC-type fasteners based on the experience of the railway line inspection staff. When the clip is completely within area A, the fastener is fastened and is in a normal state. When the clip appears in area B, the fastener is in a loosening state.

### 4.2. Classification Model

ResNet [54] is a classical deep convolutional network that is widely used in image classification, detection, and segmentation. The core of ResNet is the residual block, as shown in Figure 9. By adding a shortcut branch to the residual block, the problem of gradient disappearance caused by the increase in the number of neural network layers is effectively solved, allowing ResNet to improve the network performance by increasing the number of network layers. The output function of the residual module is as follows:

(4) $$\begin{array}{c} y=F\left(x,\left\{w_{i}\right\}\right)+x, \end{array}$$

where *x* and *y* are the input and output vectors of the residual block. *F*(*x*, {*w*_*i*_}) represents the feature vector obtained after the input vector passes through *i* convolutional layers. If the residual block has the same structure as that shown in Figure 9 and contains two weight layers, and then the formula of *F*(*x*, {*w*_*i*_}) is as follows:

(5) $$\begin{array}{c} F\left(x,\left\{w_{i}\right\}\right)=W_{2}f_{1}\left(W_{1}x+b_{1}\right)+b_{2}, \end{array}$$

where *f*_1_ is ReLU function.

Different depth ResNet models can be obtained by setting various channel numbers and residual blocks in the module. In this study, the ResNet101 model is used to detect the state of the Pandrol clip fasteners.

## 5. Experiments and Analysis

### 5.1. Data Set

The images are collected from the Shijiazhuang-Taiyuan high-speed railway line, as shown in Figure 10. The LQ-H3X industrial linear array camera, which is mounted on the special rail inspection vehicle, is used to collect the track images on the line. Through repeated image data acquisition experiments on site, high-resolution grayscale images of 2,572 track fasteners have been collected successfully, including 1,425 images of ballastless tracks and 1,147 images of ballast tracks, whose image resolutions are 4096 × 2048 pixels.

In the localization experiment on rails and fasteners, 2,572 collected original images were selected as the data set. The data set of the rail surface defect detection experiment is composed of two parts: one is derived from the rail subimage obtained from the rail and fastener localization experiment results, and the other is derived from the public rail surface discrete defect (RSDD) data set [32]. We obtained 526 images, of which rail surface has at least one defect, with width between 140 and 170 pixels and height between 600 and 700 pixels. We selected 825 subimages of fasteners from the experimental results of rail and fastener localization as the data set of fastener state detection, including 705 normal fasteners, 71 loosening fasteners, and 49 broken fasteners. As the number of loosening fasteners and broken fasteners is relatively small, data augmentation methods such as rotation, Gaussian noise, and salt-and-pepper noise are used to expand the samples of defective fasteners. Then, 705 normal fasteners, 152 loosening fasteners, and 130 broken fasteners were obtained as the data set of this experiment ultimately. Of the total number of images, 70% were randomly selected from the data set as the training set, including 494 normal fasteners, 106 loosening fasteners, and 91 broken fasteners. The remaining 30% of the images were used for testing, including 211 normal fasteners, 46 loosening fasteners, and 39 broken fasteners.

### 5.2. Experimental Environment

The experimental environment of this study is based on Windows 10, NVIDIA RTX 2080TI 11 GB GPU, Intel Xeon Silver 4214 2.2 GHz dual CPU and 64 GB RAM. The algorithm based on deep learning was developed using PyTorch framework.

### 5.3. Training Process

The overall training process of our method is shown in Figure 11, which is described as follows:

  Step 1: use LabelImg to mark the rail and fastener area in the images of original data set for the training of the improved YOLOv5s to obtain the rail and fastener localization model.
  Step 2: use the images of original data set as the input to the rail and localization model to obtain the rail subimage and the fastener subimage.
  Step 3: combine the rail subimage obtained in Step 2 with the public RSDD dataset as the rail dataset, and use LabelMe to mark the rail surface defect contours in the dataset for Mask R-CNN training to obtain rail surface defect detection model.
  Step 4: use the fastener subimage obtained in Step 2 as the fastener data set for the training of the ResNet101 model to obtain the fastener state classification model.

In the process of training the rail and fastener localization model, 2572 images were randomly assigned 1543 images as the training set, 2 257 images as the verification set, and the remaining 772 images as the test set. Due to the limitation of the performance of the GPU, the input image is resized to 1024 × 512 pixels during the training. The specific parameter settings of the model are shown in Table 1 and the loss curve of the training process is shown in Figure 12. During the first 20 epochs, training loss converges rapidly, and the decline rate of the train loss value of the model decreases. After 100 epochs, the training efficiency of the model reaches saturation loss value, and the change of loss value is small.

During the training process of the rail surface defect detection model, 526 images were randomly assigned 368 as the training set, 52 as the verification set, and the remaining 106 images as the verification set. In this experiment, the size of the image input to the training model is resized to 160 × 650 pixels. The threshold value of the intersection over union (IoU) in the RPN network was set as 0.6; that is, the IoU between the proposal and ground truth was greater than 0.6, which was retained as the positive sample. Other parameters of the model are shown in Table 2. The loss curve of the training process is shown in Figure 13. The training loss value decreases rapidly before 2500 iterations and tends to be stable after 20000 iterations, finally stabilizing at around 0.06.

### 5.4. Localization Experiment of the Rail and Fastener

#### 5.4.1. Analysis of Experimental Results

Figure 14 shows the visual detection results of two different types of track bed. According to the figure, the proposed model can realize the positioning of rails and fasteners on both ballastless and ballast railway track images.

To further verify the effectiveness of the proposed model, five object detection methods, namely, SSD [55], Faster R-CNN, YOLOv3 [56], Tiny-YOLOv3, and original YOLOv5s, were selected for comparison in this study. VGG16 [57] was used for SSD, Resnet50 was used for Faster R-CNN, and Darknet53 [56] was used for Yolov3. Precision (P), recall (R), mean average precision (mAP), and detection speed (FPS) were used as evaluation indexes for object detection:

(6) $$\begin{array}{c} \text{precision}=\frac{\text{TP}}{\text{TP}+\text{FP}}\times 100\%,\\ \text{recall}=\frac{\text{TP}}{\text{TP}+\text{FN}}\times 100\%,\\ \text{mAP}=\frac{\sum_{d=1}^{D}AP\left(d\right)}{D}, \end{array}$$

where TP, FP, and FN represent true positive, false positive, and false negative cases, respectively. AP is the area covered under the P-R curve, and *D* represents the number of categories detected. *D*=2 was used in this experiment.

The results are shown in Table 3. Detection speed of Tiny-YOLOv3 is obviously faster than that of other methods, but its detection accuracy is only 76.52%. Faster R-CNN has the best detection performance but the lowest detection speed. The detection performance of the proposed model is similar to that of Faster R-CNN and Yolov5s, but the detection speed is significantly faster than that of Faster R-CNN, which is improved by 17.52% compared with the original Yolov5s. At the same time, our model is only 12.6 M in size and can be flexibly deployed on devices with small memory. Therefore, the performance of the object detection model proposed in this study is better than that of the other five methods in our data set.

#### 5.4.2. Experiment of Rail Surface Defect Detection

Figure 15 shows the comparison results of the method proposed in this study and other methods for the detection of rail surface defects on different scales, where both PSPNet [58] and Deeplabv3+ [59] chose Resnet50 for the feature extraction network, and the boundary box was ignored for Mask R-CNN. Mask R-CNN has the best detection effect for slight defect because the addition of FPN in the backbone greatly improves the detection performance of small objects. In the three models of moderate and severe defects, the existence of defects can be detected well. However, the prediction of the defect edge by Mask R-CNN is significantly more accurate, and the defect contour can be segmented completely. In addition, the detection effect of Deeplabv3+ was also good, but the segmentation accuracy was inferior to that of Mask R-CNN. The segmentation accuracy of PSPNet was the worst, especially for the segmentation with slight and moderate defects. Therefore, the proposed method has high segmentation accuracy and robustness advantages compared with the other two methods.

To obtain quantitative experimental results, pixel accuracy (PA), mean pixel accuracy (MPA), mean intersection over union (MIoU), and frequency weighted intersection over union (FWIoU) were used as evaluation indexes in this experiment. Their specific expressions are as follows:

(7) $$\begin{array}{c} \text{PA}=\frac{\sum_{i=0}^{c}p_{ii}}{\sum_{i=0}^{c}\sum_{j=0}^{c}p_{ij}},\\ \text{MPA}=\frac{1}{c+1}\sum_{i=0}^{c}\frac{p_{ii}}{\sum_{j=0}^{c}p_{ij}},\\ \text{MIoU}=\frac{1}{c+1}\sum_{i=0}^{c}\frac{p_{ij}}{\sum_{j=0}^{c}p_{ij}+\sum_{j=0}^{c}\left(p_{ji}-p_{ii}\right)},\\ \text{FWIoU}=\frac{1}{\sum_{i=0}^{c}\sum_{j=0}^{c}p_{ij}}\sum_{i=0}^{c}\frac{p_{ii}\sum_{j=0}^{c}p_{ij}}{\sum_{j=0}^{c}p_{ij}+\sum_{j=0}^{c}\left(p_{ji}-p_{ii}\right)}, \end{array}$$

where *p*_*ij*_ represents the total number of pixels that belong to the *i* class but are predicted to be in *j*class, and *c* represents the number of categories. Two categories are used in this experiment, namely, defects and background.

Table 4 records the specific quantitative experimental comparison results. As shown in the table, the performance of PSPNet is significantly lower than that of Deeplabv3+ and Mask R-CNN in MPA and MIoU, with only 74.48% and 73.65%, respectively. The Mask R-CNN model used in this paper achieves the best results in all indicators. One of the main reasons is that Mask R-CNN is a two-stage object detection network and only segments candidate boxes generated in the first stage, which is conducive to the improvement of segmentation accuracy. Therefore, Mask R-CNN performs better in the test set of our dataset.

#### 5.4.3. Experiment of Fastener State Detection

We selected some classification models based on deep learning algorithms and some classification models based on traditional shallow learning algorithms to compare our method:

1. VGG16: a classic deep learning framework is widely used in object classification and feature extraction networks.
2. HOG + SVM: HOG feature extraction is performed on the coupler image, and then the extracted HOG feature is input to SVM for coupler status classification.
3. Canny + HOG + SVM: Canny operator [60] first extracts the edge contour features of the coupler image to obtain the edge feature map. The HOG features are extracted from the edge feature map. The SVM algorithm is used for classification finally.

The results of different classification models are shown in Table 5.  Figure 16 shows the accuracy comparison results of the various methods. The experiment shows that, compared with the other three methods, Resnet101 achieves the best detection results in our fastener data set. In addition, VGG16 and Resnet101 based on deep learning framework are significantly better than the other two methods in the detection accuracy for all types of coupler. One main reason is that VGG16 and Resnet101 extract advanced semantic features of coupler images by using the convolutional layer, while the other two methods only extract the low-level features of the image by using the artificially designed feature extraction method. Thus, they are better than the traditional machine learning method in terms of classification accuracy and robustness. Canny + HOG + SVM is better than HOG + SVM because the former method first uses a Canny operator to extract the edge features of the coupler image before extracting HOG features, so that the interference of background and other useless information is reduced on classification, and the classification precision improves to a certain extent. Compared with VGG16, Resnet101 improved the detection accuracy of loosening fasteners by 5.13% and the overall detection accuracy by 1.01%, because Resnet101 uses residual blocks to increase the depth of the CNN. This feature enables Resnet101 to have stronger feature extraction capability.

## 6. Conclusions and Future Work

This study proposed a nondestructive detection method based on deep learning algorithms to implement rail surface and fasteners defect detection. At the object localization stage, part of the structure of the backbone based on the YOLOv5 framework is improved to achieve the localization of the rail and fastener rapidly. Compared with other object detection methods, our method has the highest detection accuracy and fastest detection speed, and the model size is only 12.6 M. At the defect detection stage, Mask R-CNN is used as the defect detection model of the rail surface. Experiments show that our method is more suitable for defect detection of rail surface compared with other advanced semantic segmentation methods. In the state detection of fasteners, a set of criteria for judging the state of SFC-type fasteners is given to judge whether the fasteners are in a normal or loosening state. A comparison between the classification models based on deep learning or traditional machine learning theory can show that ResNet is the most suitable classification method for the fasteners in this data set. In general, the proposed method can effectively detect rail surface defects and fastener states.

In the future, we intend to gain more advanced knowledge of deep learning and optimize the rail surface defects detection model to improve the accuracy of defect segmentation. In our data set, few samples of rail surface defects and fastener defects are available, so we will try to use more data augmentation methods to expand the defect samples and can further improve the robustness of our method.

## Figures and Tables

**Figure 1:** Railway track line.

**Figure 2:** Overall framework of rail surface and fastener defect detection method.

**Figure 3:** Improved YOLOv5 network.

**Figure 4:** Backbone before and after improvements.

**Figure 5:** Ghost bottleneck.

**Figure 6:** Rail surface defect detection model.

**Figure 7:** Different types of SFC fastener state. (a) Normal. (b) Loosening. (c) Broken.

**Figure 8:** Division of the fastener state judgment area.

**Figure 9:** Residual block.

**Figure 10:** Image acquisition. (a) Picture of image acquisition in Shijiazhuang-Taiyuan high-speed railway line. (b) Special rail inspection vehicle.

**Figure 11:** Overall training process.

**Figure 12:** Training loss curve of the rail and fastener localization model.

**Figure 13:** Training loss curve of the rail surface defect detection model.

**Figure 14:** Visualization results of rail and fastener localization. (a) Ballastless track image. (b) Ballast track image.

**Figure 15:** Comparison of detection results of rail surface defects with different methods: (a) original image, (b) ground truth, (c) PSPNet, (d) Deeplabv3+, and (e) Mask R-CNN.

**Figure 16:** Accuracy of different fastener state classification models.

**Table 1:** Parameters of rail and fastener localization model.

Parameters	Value
Input size	1024 × 512
Initial learning rate	0.01
Class	2
Batch size	6
Epochs	120

**Table 2:** Parameters of the rail surface defect detection model.

Parameters	Value
Learning rate	0.001
Weight decay	0.0001
Batch size	4
Class	1
Iterations	30000

**Table 3:** Comparison of different object detection methods.

Method	P (%)	R (%)	mAP (%)	Model size (MB)	FPS
SSD	94.72	99.73	98.96	181.2	61.3
Faster R-CNN	97.12	100	99.76	267.8	12.2
YOLOv3	96.81	99.73	99.74	117.2	62.5
Tiny-YOLOv3	76.52	98.04	92.92	16.6	168.4
YOLOv5s	96.41	100	99.71	14.1	83.3
Ours	96.23	100	99.68	12.6	97.9

**Table 4:** Comparison of different segmentation models.

Method	PA (%)	MPA (%)	MIoU (%)	FWIoU (%)
PSPNet	99.41	74.48	73.65	98.84
Deeplabv3+	99.65	92.76	85.67	99.38
Mask R-CNN	99.72	94.37	87.52	99.51

**Table 5:** Classification results of different classification models.

Method	Normal fastener	Loosening fastener	Broken fastener
HOG + SVM	206/211	37/46	31/39
Canny + HOG + SVM	208/211	40/46	32/39
VGG16	211/211	44/46	34/39
ResNet101	211/211	45/46	36/39

## Data Availability

The data used to support the findings of this study are available from the corresponding author upon request.
